RETRACTED

# Comparison of Challenges and Problems Encountered in the Practice of Exclusive Breast Feeding by Primiparous and Multiparous Women in Rural Areas of Sindh, Pakistan: A Cross-Sectional Study

**DOI:** 10.7759/cureus.14976

**Published:** 2021-05-12

**Authors:** Sana Zafar, Khizer Shamim, Syeda Mehwish, Mohsin Arshad, Rahil Barkat

**Affiliations:** 1 Biological Sciences, Victoria University of Wellington, School of Biological Sciences, Wellington, NZL; 2 Medicine, Ziauddin Hospital, Karachi, PAK; 3 Dentistry, Karachi Medical and Dental College, Karachi, PAK; 4 Department of Internal Medicine, Multan Medical and Dental College, Karachi, PAK; 5 Indus Hospital Research Center, The Indus Hospital, Karachi, PAK

**Keywords:** challenges, exclusive breastfeeding, practice, primiparous, multiparous

## Abstract

Introduction: The UNICEF (United Nations International Children Education Fund) and WHO (World Health Organization) recommend exclusive breastfeeding (EBF) for the first six months of life. EBF is considered to be an important practice for enhancing infant health and wellbeing. Breastfeeding offers a wide range of psychological and physical health benefits in the long-term and short-term for young children, infants, and mothers. This study aims to compare exclusive breastfeeding practice among primiparous and multiparous mothers including reasons for discontinuing exclusive breastfeeding and problems faced during breastfeeding.

Methodology: This cross-sectional study was conducted in rural areas of Sindh, registered with the Maternal Newborn Health Registry (MNHR). The study used a systematic sampling technique for the enrollment of study participants. A survey questionnaire was used to collect data from mothers about the practices of EBF. A total of 397 mothers were interviewed and analyzed.

Results: Among Primiparous mothers, 14.1% of mothers initiated breastfeeding within one hour of birth, while 22.4% of multiparous mothers, initiated breastfeeding within one hour of birth. The difference between the two is statistically insignificant (p-value=0.234). A high percentage of multiparous mothers exclusively breastfed their infants for six months (63.5%) as compared to primiparous mothers (51.5%). The most common reason for introducing pre-lacteal feed before six months among primiparous mothers is the lack of adequate milk production to fulfill baby needs; this was the case for 35.4% of mothers. On the other hand, the baby remaining hungry post breastfeeding was the major reason among multiparous mothers (44.0%) for introducing pre-lacteal feed before six months.

Conclusion: This study helped in the identification of issues faced by primiparous and multiparous mothers during exclusive breastfeeding. Interventions for promoting EBF need to be tailored as per the need and challenges of the population.

RETRACTED

## Introduction

The UNICEF (United Nations International Children Education Fund) and WHO (World Health Organization) recommend exclusive breastfeeding (EBF) for the first six months of life [1]. EBF is defined as feeding infants only breast milk and no other drink or food, not even water, for the first six months of life. However, infants are allowed to receive medicines, minerals, and vitamins [2]. EBF is considered to be an important practice for infants to enhance their health and wellbeing [3]. Breastfeeding offers a wide range of psychological and physical health benefits in the long-term and short-term for young children, infants, and mothers. Breastfeeding is associated with a lower risk of diabetes, obesity, atopic dermatitis, gastroenteritis, otitis media, asthma, and respiratory infections among infants. Benefits of exclusive breastfeeding for mothers include reduced risk of ovarian cancer, breast cancer, and postpartum depression [4].

Despite such tremendous potential and extensive programs to encourage breastfeeding around the world, the 2017 Global Breastfeeding Scorecard, which analyzed 194 countries, revealed surprisingly low scores. According to the survey, only 40% of children under the age of six months receive EBF on a global scale. At most, 23 of the 194 countries had EBF rates of more than 60%, with rates of continued breastfeeding up to the age of one year hovering around 74% [5]. In Pakistan, only 48% of infants are exclusively breastfed during the first six months of their life [6]. Despite seeing an increase in the rate of EBF over the last five years, Pakistan has the second-lowest EBF rate among all South Asian countries [7].

Primigravida mothers are considered to be a vulnerable group where the provision of inadequate or inaccurate messages can lead to reduced chances of initiating EBF [8]. Primigravida mothers are more prone to accepting non-scientific health promotional messages received through different sources [7]. Primiparous mothers when compared to multiparous mothers are more likely to face challenges in practicing exclusive breastfeeding. They are more likely to experience difficulties when adjusting to a new role and with low breastfeeding skills [9]. There is a need and requirement for multidimensional interventions that concomitantly tackle various aspects of breastfeeding barriers and problems in order to efficiently enhance rates of breastfeeding.

Low rates of breastfeeding during the first six months suggest that mothers constantly face several barriers to continue breastfeeding [10]. The early postpartum period is considered to be a critical period for establishing and supporting breastfeeding. Previous studies conducted in Sindh, Pakistan reported factors contributing toward the practice of EBF among mothers but to the best of our knowledge, no study was carried out in Sindh, that identified and compared challenges and problems among primiparous and multiparous mothers. Identifying challenges can help policymakers and healthcare professionals to design interventions and strategies that can help mothers overcome issues faced during breastfeeding. This will enhance the practice of exclusive breastfeeding among mothers in Sindh, Pakistan. This study aims to compare exclusive breastfeeding practices among primiparous and multiparous mothers including reasons for discontinuing exclusive breastfeeding and problems faced during breastfeeding.

RETRACTED

## Materials and methods

Study design and study setting

This cross-sectional study was conducted in rural areas of Sindh, registered with MNHR (Maternal and Neonatal Health Registry). MNHR is a population-based study for low- and middle-income countries (LMICs) to assess pregnancy-related outcomes. In MNHR, two sub-districts of Thatta are divided into eight clusters, including urban and rural areas, and the survey was implemented in all eight clusters. Thatta is one of the largest cities in Sindh, Pakistan. The major livelihood activity among the people of Thatta is agriculture. Despite its proximity to major urban cities such as Karachi, Thatta was ranked 64 out of 91 districts in Pakistan on the Human Development Index in 2003. According to recent estimates, the region lags behind other parts of the country in terms of education, health, and jobs. It has the lowest educational attainment rate in the Sindh province. It is one of Pakistan's five worst-performing districts of Sindh.

Eligibility criteria

All mothers included having a baby of 6-12 months of age at the time of enrollment and who were ready to be a part of the study. All mothers who had a disease due to which breastfeeding was contraindicated or not possible were excluded. Besides this, mothers who had a baby with a condition at the time of birth in which breastfeeding was contraindicated were also excluded.

Sample size and sampling technique

The sample size was calculated using OpenEpi Software for estimation of single population proportion assuming prevalence for exclusive breastfeeding in Pakistan is 48%, confidence limit of 5%, design effect of 1.0, and non-response rate of 5%. The total sample size calculated was 403. Mothers were recruited into this study using systematic random sampling. A list of all mothers having a 6-12 months old baby at the time of the study period was obtained from MNHR. Households of selected mothers were visited for data collection. In case if a mother did not give consent or excluded from the study, a mother present next to that mother in the list was interviewed for data collection.

RETRACTED

Data collection

Data were collected using a survey questionnaire that was composed of three sections. Section 1 assessed the sociodemographic characteristics of mothers including the age of the mother, educational status of the mother, total household income, gender of the child, and mother occupation. Section 2 of the survey questionnaire included the details about the place of birth of the indexed child, the person who attended the delivery, how soon mother started the breastfeeding after birth, antenatal care, and gestational age of the baby. The last section of the questionnaire was about the problems faced by mothers during breastfeeding and reasons for discontinuing breastfeeding.

The dependent variable in this study was the prevalence of exclusive breastfeeding till six months among primiparous and multiparous mothers who were assessed by asking the question “Did they introduced any food or liquid item in baby’s diet before six months of the birth other than medicines and vitamins?” from mothers. The primary group variable was the maternal parity that was categorized into two groups primiparous and multiparous.

Ethical consideration

Approval for this study was taken from IRB (Institutional Review Board) of The Indus Hospital. Verbal consent was taken from participants before enrollment.

Data analysis

The data were checked, cleaned, coded, and analyzed using STATA software version 16.0 (StataCorp LP, College Station, TX). Descriptive statistics such as mean, standard deviation, frequency, and percentage were computed to describe socio-demographic characteristics, the prevalence of exclusive breastfeeding, frequency of mothers who initiated breastfeeding within the first hour of birth, and problems faced by mothers. The normality of continuous data was assessed using the Shapiro-Wilk test, skewness, and kurtosis. Comparison of continuous and categorical variables between primiparous and multiparous mothers were done by using a t-test and chi-square test of independence respectively. A P-value of less than or equal to 0.05 was considered significant.

## Results

A total sample of 397 mothers was selected and analyzed from the survey conducted in rural areas of Sindh, Pakistan. Demographic characteristics of mothers and infants were collected. A total of 397 mothers were included in the analysis. Mothers and infants were categorized as per socio-demographic variables, such as mother’s age, education, occupation, child’s gender, and gestational age. Table 1 shows the sociodemographic characteristics of mothers and infants. Out of 398, the majority of mothers were multiparous (75.1%). The mean age of mothers in multiparous mothers (29.1±4.5) is significantly higher as compared to primiparous mothers (23.4±3.4). The majority of mothers in both groups did not attend any formal education as shown in Table 1.

RETRACTED

**Table 1:** Demographic characteristics of mothers. ^Mean (SD). *Significant at 0.05.

Variable	Primiparous mothers, n (%)	Multiparous mothers, n (%)	P-value
Age^^^	23.4 (±3.4)	29.1 (±4.5)	0.001^*^
Mother education			
Illiterate	66 (66.7)	240 (80.3)	0.005^*^
Literate	33 (33.3)	59 (19.7)	
Mother occupation			
Employed	50 (50.5)	174 (58.2)	0.181
Unemployed	49 (49.5)	125 (41.8)	
Gender of child			
Male	48 (48.5)	172 (57.5)	0.117
Female	51 (51.5)	127 (42.8)	
Gestational age			
Term baby	66 (66.7)	185 (61.9)	0.392
Pre-term/post-term baby	33 (33.3)	114 (38.1)	
Mode of delivery			
Normal	215 (63.8)	36 (59.0)	0.476
Assisted	122 (36.2)	25 (41.0)	
The person who attended the delivery			
Physician	47 (47.5)	84 (28.1)	0.001^*^
Nurse/LHV/midwife	35 (35.3)	110 (36.8)	
TBA	17 (17.2)	105 (35.1)	
Antenatal care			
Yes	98 (99.0)	280 (93.6)	0.035^*^
No	1 (1.0)	19 (6.4)	

Early infant feeding practices

The majority of multiparous and primiparous mothers did not initiate breastfeeding within the first hour of delivery. Among primiparous mothers, 14.1% of mothers initiated breastfeeding within one hour, while 22.4% of multiparous mothers initiated breastfeeding within one hour, and the difference is statistically insignificant (p-value=0.234). A high percentage of multiparous mothers exclusively breastfed their infants for six months (63.5%) as compared to primiparous mothers (51.5%). There is a significant difference in the prevalence of exclusive breastfeeding between multiparous and primiparous mothers showing the association between parity and exclusive breastfeeding rate in this study population as shown in Table 2.

**Table 2:** Frequency of early initiation and exclusive breastfeeding among primiparous and multiparous mothers. *Significant at 0.05.

Variable	Primiparous mothers, n (%)	Multiparous mothers, n (%)	P-value
Initiation of breastfeeding within one hour			
Within one hour	14 (14.1)	67 (22.4)	0.234
After one hour	85 (85.9)	232 (77.6)	
Exclusive breastfeeding till six months			
No	48 (48.5)	109 (36.5)	0.034^*^
Yes	51 (51.5)	190 (63.5)	

Problems faced by mothers during exclusive breastfeeding

Over 21.4% and 20.4% of primiparous and multiparous mothers, respectively, reported that they faced problems during breastfeeding within the first six months. The most common problem faced by both primiparous mothers and multiparous mothers was inadequate milk production, i.e., 47.6% and 59.0%, respectively. Other problems faced by mothers during breastfeeding included a baby’s refusal to breastfeed, pain in the breast, and illness in mothers. However, no statistical difference was found between primiparous and multiparous mothers in problems faced as shown in Table 3.

RETRACTED

**Table 3:** Problems faced by mothers during exclusive breastfeeding.

	Primiparous mothers, n (%)	Multiparous mothers, n (%)	P-value
Problems faced during breastfeeding			
Yes	21 (21.2)	61 (20.4)	0.863
No	78 (78.8)	238 (79.6)	
Inadequate milk production			
Yes	10 (47.6)	36 (59.0)	0.600
No	11 (52.4)	25 (41.0)	
Baby refused to breastfeed			
No	94 (76.2)	52 (85.2)	0.339
Yes	5 (23.8)	9 (14.8)	
Pain in breast			
No	96 (85.7)	50 (81.9)	0.761
Yes	3 (14.3)	11 (18.1)	
Illness to mother			
No	96 (85.7)	54 (88.5)	0.454
Yes	3 (14.3)	7 (11.5)	

Reasons for introducing pre-lacteal food before six months of birth

Table 4 shows the reasons why nulliparous and multiparous mothers introduced pre-lacteal feed before six months. The most common reason among primiparous mothers is the lack of production of adequate breastmilk to fulfill the baby’s needs. This was found in 35.4% of primiparous mothers which was followed by 31.2% of primiparous mothers reporting that baby remained hungry after breastfeeding. On the other hand, a baby remaining hungry after breastfeeding was the major reason among multiparous mothers (44.0%) for introducing pre-lacteal feed before six months. Moreover, the production of insufficient breastmilk is the second major reason for introducing pre-lacteal feed that was reported by 28.4% of multiparous mothers.

**Table 4:** Reasons for introducing pre-lacteal food before six months of birth.

Reasons for introducing pre-lacteal food	Primiparous mothers, n (%)	Multiparous mothers, n (%)
The baby remained hungry after breastfeeding	15 (31.25)	48 (44.0)
Not producing enough milk to satisfy baby needs	17 (35.4)	31 (28.4)
Advised by relatives/friends/neighbors	9 (18.7)	19 (17.4)
Advised by healthcare providers/TBA	9 (18.7)	11 (10.1)
Others	4 (8.3)	10 (9.2)

## Discussion

In a developing country such as Pakistan, breastfeeding not only comes as a natural means to feed the infant but also helps decrease the economic burden for the parents. Other than that, there are several health benefits to breastfeed an infant for the first six months, one of which is decreased incidence of diarrhea in the children who are preferably breastfed exclusively [11]. Our study focuses on the challenges faced by the primiparous mothers compared to the multiparous mothers in maintaining EBF for six months postpartum.

RETRACTED

Though a necessity, breastfeeding an infant exclusively for six months may present a number of challenges for mothers especially in a rural dwelling with limited resources. Out of several, one challenge that came out significantly in our study was unsupportive family members. For both, primiparous and multiparous mothers, family support was found to be positively related to exclusive breastfeeding for up to six months after delivery. This is in line with a study conducted in Ethiopia, where living in joint families aided the mothers to continue breastfeeding for longer [12]. The reason being extra support; financial, physical as well as emotional support from the family help the mother to continue EBF for six months.

Another factor showing a positive impact on EBF for the first six months was the age of the mother. According to our data, multiparous mothers were older than primiparous, and they breastfed their infants more exclusively for the first six months of life. This finding is in line with the study conducted in Kenya comparing the breastfeeding behaviors of primiparous and multiparous mothers. They found that multiparous mothers exclusively breastfed their babies more (49.3%) than primiparous (39.5%) [2].

A study conducted in Brazilian rural areas deduced how antenatal care and the availability of healthcare facilities aids in exclusive breastfeeding behaviors in women [13]. The study highlighted that if these women, primiparous or multiparous, have an access to proper care and knowledge of breastfeeding and its advantages, they would opt for it. Women with sound knowledge and facts regarding the practice of EBF including its impact on the lives of the mother and the child were seen more to practice the action for six months after delivering their child. This finding is similar to our study where the provision of antenatal care was statistically significant, suggesting that their knowledge of the importance of EBF as well as the care given to them while pregnant contributed to the prevalence of the practice for a longer period of time.

An important factor was the literacy of the mothers taking part in the study. Though the majority of the participants were illiterate be it primiparous (66.67%) or multiparous (80.27%), and none of them had received any formal education on the matter, a certain percentage for primiparous (33.33%) and multiparous (19.73) were counted as literate. Their knowledge of breastfeeding, its benefits and positive outcomes on the mother’s and child’s life might be the contributing factor to be positively impacting exclusive breastfeeding behaviors in mothers. The findings are in line with several studies which also reiterated the similar consequences of literacy and exclusive breastfeeding [13,14].

RETRACTED

It was found that mothers with higher education were not much prone to continue breastfeeding their infant until the age of six months. However, those with comparatively lesser education or illiteracy were more inclined to exclusively breastfeed their children for a longer period of time. This finding was in line with another study conducted in the rural areas of Tamil Nadu, India. There the mothers who studied past matriculation were more prone to stop breastfeeding before their child turned six months, while those who had studied till matriculation or less were more in favor of exclusive breastfeeding for six months or more postpartum [15].

Though it is suggested for the mothers and the child to observe exclusive breastfeeding for at least the first six months of life, several reasons were identified which contributed to the introduction of lacteal diet in infants. The most common was the baby remaining hungry after feeding which could be due to insufficient milk production. Women facing this issue turned toward pre-lacteal diets as they would aid with the problem while keeping the baby healthy. Other reasons included advice to change the baby’s diet by the relatives or the healthcare professional. The findings were in line with an Iranian study that focused on the reasons why mothers would not exclusively breastfeed their infants for the first six months after being born. Out of the reasons identified, the advice of the healthcare professional and lack of milk production were among the first two reasons for introducing an early pre-lacteal diet [16].

Our study was one of the very few studies conducted in the rural areas of Pakistan. The issues highlighted in the study remain a jarring dilemma in countless households with scarce means to get by, as the lack of knowledge regarding breastfeeding adds insult to the injury. For the health of the mother and the child, it is imperative to maintain the practice of breastfeeding as advised by most of the healthcare professionals, however, in deprived areas of the country, it becomes a luxury to have such essential knowledge.

The study has certain limitations including the limitations of the study design used, i.e., cross-sectional study. The study might include recall bias as only mothers with babies of 6 to 12 months of age were included in the study. Second, the study was not complemented with qualitative data due to which understanding about cultural and nutritional impacts on exclusive breastfeeding will not be accomplished.

RETRACTED

## Conclusions

The study has shown that the prevalence of exclusive breastfeeding is different in multiparous and primiparous mothers. The findings of our study have shown that challenges during breastfeeding are the same among primiparous and multiparous mothers of our study population. Interventions for promoting EBF need to be tailored as per the need of the population. Efforts for promoting EBF need to focus on enhancing the knowledge and attitude of mothers and preparing them to face challenges. It is also important to consider factors while planning and implementing strategies to promote EBF. The findings of our study will be useful particularly to those organizations that focus on behavior change communication interventions to improve EBF.
